This article has been retracted.

# DNA Damage Response Genes in Osteosarcoma

**DOI:** 10.1155/2021/9365953

**Published:** 2021-11-02

**Authors:** Ying Tang, Yan-xia Liu, Xiuning Huang, Peng Li

**Affiliations:** ^1^Trauma Center, State Key Laboratory of Trauma, Burns and Combined Injury, Institute of Surgery Research, Daping Hospital, Army Medical University, No. 10 Changjiang Zhi Road, Yuzhong District, Chong Qing 400042, China; ^2^Department of Pharmacognosy and Traditional Chinese Medicine, College of Pharmacy and Laboratory Medicine, Army Medical University, No. 30 Gaotanyan Centre Street, Shapingba District, Chong Qing 400038, China

## Abstract

**Background:**

Improving the osteosarcoma (OS) patients' survival has long been a challenge, even though the disease's treatment is on the verge of progress. DNA damage response (DDR) has traditionally been associated with carcinogenesis, tumor growth, and genomic instability. No study has used DDR genes as a signature to identify the prognosis of OS. The goal of this work was to find an effective possible DDR gene biomarker for predicting OS prognosis, which may be useful in clinical diagnosis and therapy.

**Methods:**

To assess gene methylation, univariate and multivariate cox regression analyses were performed on data from OS patients. The data were retrieved from public databases, including the Therapeutically Applicable Research to Generate Effective Treatments (TARGET) and the Gene Expression Omnibus (GEO).

**Results:**

The DDR gene signature was chosen, which included seven genes (NHEJ1, RMI2, SWI5, ERCC2, CLK2, POLG, and MLH1). In the TARGET dataset, patients were categorized into two groups: high-risk and low-risk. Patients with a high-risk score revealed a shorter OS rate (hazard ratio (HR): 3.15, 95% confidence interval (CI): 1.38–4.34, *P* < 0.001) in comparison with the patients with a low-risk score in the TARGET as a training group. The validation of the prognostic signature accuracy was carried out in relapse and validation cohorts (TARGET, *n* = 75; GSE21257, *n* = 53). The signature was found to be an independent predictive factor for OS in multivariate cox regression analysis, and a nomogram model was developed to predict an individual's risk of OS. DDR gene signature involved in Fanconi anemia pathway, nonhomologous end−joining pathway, mismatch repair, and nucleotide excision repair pathway.

**Conclusions:**

Our study suggests that the identified novel DDR genes could be a powerful prognostic tool for prognosis evaluation and a valuable tool in predicting the risk factors in OS patients.

## 1. Introduction

The most common primary malignant tumour of bone is osteosarcoma, which occurs most frequently in teens and young adults during the pubertal growth spurt [1]. Despite advancements in chemotherapy, surgery, and radiotherapy, patients with osteosarcoma without metastases have a 5-year OS rate of 78% [2]. OS, on the other hand, still has a 30% mortality rate [3]. Even though numerous ways for diagnosing and treating osteosarcoma have been established, new approaches for the treatment and prevention are required to be developed. The pathophysiology of osteosarcoma progression is still a mystery. As a result, finding efficient diagnostic markers and researching the leading molecular etiology of osteosarcoma is critical.

In many solid tumors, defective alterations during DNA repair can result in a significant increase in the frequency of neoantigens [4]. As a result, poor DNA repair has been linked to better clinical responses to PD-1 inhibition. A weakened mismatch repair (MMR) gave better therapeutic benefits with pembrolizumab in individuals with colorectal cancer [5–7] and the study of various solid tumors [8]. These findings have led to the FDA's landmark approval of PD-1 inhibitors in MMR-deficient malignancies, signaling a paradigm shift toward oncologic therapy based on molecular proficiency [8]. Several different DNA repair mechanisms have been linked to the accumulation of neoantigens. In a study of patients with NSCLC, POLE, MSH2, and mutations in POLD1 were found in excessive tumor neoantigens burden, which was linked to enhanced PD-1 treatment responsiveness. Additionally, polymerase epsilon (POLE) mutations in endometrial cancers had higher expression of neoantigen burden and PD-L1 [9], and these mutations have been linked to exceptional immunotherapy responders [10]. Changes in the homologous recombination apparatus including BRCA2 and BCRA1 mutations were also linked to increased neoantigen load and overall survival following the treatment with anti-PD-1 [11]. Somatic alterations affecting the DNA damage repair (DDR) pathways and/or cell cycle are found in multiple subsets of osteosarcomas, and clinical trials are being designed to test precision medicine approaches based on these aberrations. However, the biomarker of DDR genes in the prognosis of OS has not yet been explored.

In the current study, we have examined and validated candidate DNA damage repair signature as a marker to predict prognosis by utilizing the GEO and TARGET databases. Identification of DNA damage repair signature will allow patients to be separated into low-risk and high-risk groups. Moreover, the expression pattern of DDR genes could be used as an independent prognostic signature for OS patients, allowing for the development of new treatment targets and diagnostic biomarkers.

## 2. Materials and Methods

### 2.1. Dataset and Data Processing

The data generated by the OS project of the TARGET (https://ocg.cancer.gov/programs/target) were used as the training set. The TARGET osteosarcoma project was used for the important clinical information for osteosarcoma patients as well as level three RNA-Seq data. As a validation set, the GEO dataset GSE21257 was employed. The GEO database was used for collecting the survival information of dataset GSE21257 and mRNA data.

### 2.2. Screening of Survival-Related DDR Genes

The model was developed by employing the machine learning approach and statistics as described previously [12]. To analyze the link between the survival time, and statue, and the expression of each DDR gene in the training cohorts, the univariate cox proportional hazard regression analysis was used on the basis of earlier studies. To build a prognosis model, multivariate cox regression analysis was used to filter for the most powerful and reliable predictive prognostic methylation sites. On the basis of the model, the prognosis risk was calculated using the expression equation as follows:

(1) $$\begin{array}{c} \text{risk score}\left(\text{RS}\right)=\sum_{i=1}^{N}{\text{Exp}}_{i}*{\text{Coef}}_{i}, \end{array}$$

the number of expression of DDR gene signature is indicated by *N*, the expression of the DDR genesis is indicated by Exp_*i*_, and multivariate cox regression coefficient is indicated by Coef_*i*_. The risk score (RS) was the multinode weighted sum of risk scores, calculated using the signature coefficient for each patient as reported earlier. The median risk score was utilized as the cutoff value for dividing the training, test, and validation cohorts into high- and low-risk groups. The log-rank test was employed for comparing the prognoses between two groups using Kaplan–Meier (K–M) survival analysis. The independent survival prediction of the methylation fingerprints was investigated via multivariable cox regression analysis. The methylation genes and differential expression between surrounding tissues and tumors were screened using the Student's *t*-test.

### 2.3. Functional Enrichment Analyses

The pathway enrichment analysis was carried out for the genes on the basis of the Gene Ontology (GO) database (biological process, cellular component, and molecular function abbreviated as BP, CC, and MF, respectively) and Kyoto Encyclopedia of Genes and Genomes (KEGG). For multiple comparisons, the *P* values were adjusted using the false-discovery rate (FDR) approach. The R package clusterProfiler was used to conduct all of the analyses [13].

### 2.4. Construction of the Nomogram

A nomogram was developed incorporating the two independent clinical risk factors (metastasis and age) and the methylation sites signature to predict the 1-, 3-, and 5-year survival rate in clinical practice. On a point scale, the nomogram score was determined for each variable. Following the calculation of the overall nomogram score, we calculated the anticipated 1-, 3-, and 5-year survival rates for each patient, as previously discussed.

### 2.5. Statistical Evaluations

The statistical evaluations were carried out with R 3.5.1 (https://www.r-project.org). pROC and Bioconductor (https://bioconductor.org) were used for downloading all the survivals. The two-tailed *t*-test with Mann–Whitney *U*-test was employed to identify the statistical variations between the two groups. A threshold *P* value <0.05 was regarded as statistically considerable for different analyses and correlations. The Wilcoxon rank-sum test was employed to determine the significance of the comparisons, and the results are displayed as mean *P* values (^*∗∗*^*P* < 0.01; ^*∗∗*^*P* < 0.05).

## 3. Results

### 3.1. Evaluation of the Prognostic DDR Genes from the Training Cohort

We first obtained DDR genes list from the study of Knijnenburg et al., [2], and then we integrated the expression of DDR genes in TARGET database samples. The sample from the TARGET database as the training group, with complete clinical information, was used for collecting more information on the association of prognosis with 276 genes. Being the independent variables, the survival statue and survival time were initially conducted using univariate cox proportional hazards regression analysis of the 276 genes. 18 DDR genes were considerably linked with the patients prognosis (*P* < 0.05; Figure 1(a) and Table S1). Furthermore, to obtain the highly predictive prognostic DDR genes, a multivariate cox regression analysis was carried out for the seven identified DDR genes set (NHEJ1, RMI2, SWI5, ERCC2, CLK2, POLG, and MLH1, Figure 1(b)) model to evaluate the prognosis risks for the patients. The risk score of the combination composed of NHEJ1, RMI2, SWI5, ERCC2, CLK2, POLG, and MLH1 (Table S2) was determined as follows:

(2) $$\begin{array}{c} \text{RS}=\left(0.061\times {\text{Exp}}_{\text{NHEJ}1}\right)+\left(0.06\times {\text{Exp}}_{\text{RMI}2}\right)+\left(-0.022\times {\text{Exp}}_{\text{SMI}5}\right)\\ +\left(-0.096\times {\text{Exp}}_{\text{ERRC}2}\right)+\left(0.029\times {\text{Exp}}_{\text{CLK}2}\right)\\ +\left(0.007\times {\text{Exp}}_{\text{POLG}}\right)+\left(-0.07\times {\text{Exp}}_{\text{MLH}1}\right). \end{array}$$

RS and Exp are the risk score and the expression value.

### 3.2. Confirmation of the Survival Status of the DDR Genes Signature in the TARGET Group

DDR genes signature was calculated in the risk score of all patients. To divide the training cohorts into high- (*n* = 48) and low-risk (*n* = 47) groups, the median risk score was used as the cutoff criterion. The survival rates were obtained using the K–M survival analysis. The low-risk scores patients had a 5-year survival rate of more than 75%, compared to less than 25% for the high-risk scores patients (HR: 3.15, 95% CI:1.38–4.34, *P* < 0.001, Figure 2(a)). The receiver operating characteristic (ROC) curve was utilized to identify the prognostic model's accuracy. The model's ability to predict OS patients' prognosis improves as the area under the ROC curve increases. The prognostic signature's prediction precision was reliable in the training dataset (AUC Signature **=** 0.75, Figure 2(b)). Our results demonstrate that the DDR genes signature can be a potential novel and powerful accurate prognosis biomarker.

### 3.3. Confirmation of DDR Genes Signature's Ability to Survive in the Relapse Group

We collated relapse samples and follow-up data from the TARGET database. The relapse cohorts were classified into 39 (52%) high-risk and 36 (48%) low-risk groups using the established prognostic model. In the test group, the 5-year OS was more than 75% for the low-risk group and less than 25% for the high-risk group (HR: 2.65, 95% CI: 1.43–1.79; *P* < 0.001, Figure 2(c)).

### 3.4. The Robust DDR Gene Profile Validated in Different Validation Cohorts

The signature in GSE21257 was examined for the prognosis of OS patients to validate that the found seven DDR gene-based classifiers had equal predictive value in various patients. Employing the established coefficient of the module, the training cohorts were categorized into LR group (26 (49.1%)) and HR group (27 (50.9%)). The corresponding 5‐year OS was 65% for the LR group and less than 50% for the HR group in GSE21257 (Figure 2(d)). The validation dataset also showed that the DDR gene profile used in this study was a reliable prognostic indicator.

### 3.5. Independent Prognostic Indicators and the Nomogram Development for Predicting the Prognosis of Patients

Multivariate cox regression analysis was carried out to evaluate the association between clinicopathological features (metastasis and age) and the signature risk score. In the training dataset, the association showed that the signature independently predicted the survival rate of patients (high- vs. low-risk group, HR = 0.15, 95% CI: 0.068–0.034, *P* < 0.001, Figure 3(a)). A nomogram incorporating the two clinical risk variables (metastasis and age) and the DDR genes signature was developed for predicting the 1-, 2-, and 5-year survival rates in clinical practice. According to the point scale, the tool may calculate a nomogram score for each variable. We calculated the estimated probability of 1-, 3-, and 5-year survival for each patient after computing the overall nomogram score. The signature contributed the most to the 1-, 3-, and 5-year prognosis, according to the nomogram, followed by age and stage (Figure 3(b)).

### 3.6. Functional Prediction of DDR Signature Genes

The possible participation of the DDR signature genes in biological processes involved with osteosarcoma development was investigated using GO and KEGG analyses. The functional analysis was performed with these genes. The GO findings showed that the DDR signature genes were related to DNA recombination, chromosome segregation, double-strand break repair, and nonrecombinational repair (Figure 4(a)). We also found that DDR signature genes were involved in the Fanconi anemia pathway, NHEJ pathway, mismatch repair, and nucleotide excision repair pathway (Figure 4(b)) which is essential in single or double strands of DNA and their repair systems.

## 4. Discussion

One of the most common malignant tumors in the orthopedic area is osteosarcoma. It has been invasive, has a high rate of metastatic spread, and has a bad prognosis [14]. For OS patients, the absence of appropriate prognostic indicators has been the main concern. Somatic changes impacting the DDR pathways and/or cell cycle have been seen in multiple subsets of osteosarcomas, and clinical trials are being designed to test precision medicine strategies based on these aberrations. However, more precise DDR genes signatures and stable modules to predict prognosis is needed, which can make the individualized therapeutic decision for patients with OS patients. So, we are the first to study DDR-related prognosis signature in OS patients.

In our study, we evaluated 276 DDR genes from previous research which had opposite differential expressed patterns. By applying different statistical approaches, we identified seven DDR genes signature. Furthermore, we validated the DDR genes signature in the relapse group and external validation group which is a powerful tool in predicting the prognosis and was independently associated with the overall survival for OS patients. Finally, we established a DDR signature gene nomogram to predict prognosis. We found that DDR signature genes took part in the Fanconi anemia pathway, NHEJ cascades, mismatch repair, and nucleotide excision repair pathway. Our study implicates applications in precision therapy and then eventually leads to an enhancement in the prognosis of OS patients.

We determined a set of seven DDR genes consisting of NHEJ1, RMI2, and SWI5, ERCC2, CLK2, POLG, and MLH1 that predicts prognosis in two patient cohorts.

In colorectal cancer patients, the *MLH1* gene, like a number of other suppressor genes, is susceptible to being silenced by promoter methylation [15] and, for patients with stage II and III colorectal cancer, MLH1 expression gives useful prognostic information [16]. ERCC2 is a key component of the nucleotide excision repair process, as well as cell cycle and apoptosis control and transcription initiation [17]. In colorectal and gastric cancers, ERCC2 polymorphism predicts the clinical outcomes of oxaliplatin-based chemotherapies [18]. POLG is the sole DNA polymerase found in human mitochondria, and it is required for DNA repair and replication [19]. POLG gene was considerably linked with the prognosis of hepatocellular carcinoma patients in a dose-dependent manner [20]. In breast cancer, CLK2, a kinase that phosphorylates SR proteins implicated in splicing, functions as an oncogene [21], and highly expressed CLK2 significantly enhances the proliferation of lung cancer cells, thereby promoting the occurrence and development of lung cancer [22].

In human cells, the nonhomologous end joining (NHEJ) DNA damage repair pathway is the most common pathway for DNA double-strand repair, and its abnormal activity has been linked to treatment resistance in a variety of cancers [23]. NHEJ1 deficiencies may facilitate the accumulation of mutations in the setting of DNA mismatch repair deficiency in cancers [24]. RMI2 is an important component of the BLM-TopoIIIa-RMI1-RMI2 complex, which helps to keep the genome stable [25]. RMI2 expression was linked to a poor prognosis and shorter survival time in patients with hepatocellular cancer [26] and is also important for lung cancer metastasis and growth [27]. SWI5 facilitates the Rad51-dependent recombination repair cascade and is a component of the SWI5-SFR1 heterodimers [28]. In both sporadic and familial breast cancer patients, SWI5 proteins implicated in DNA damage response were expressed [29].

Taken together, we successfully obtained prognostic signatures which may predict the survival rate of OS patients. Importantly, we developed a seven‐DDR gene nomogram to predict patients' prognosis. Our findings show that this signature has the potential to be a precise and reliable biomarker for predicting prognosis and tailoring therapy for OS patients.

## Figures and Tables

**Figure 1:** Develop DDR gene signature. (a) Univariate cox proportional hazards regression analysis of the DDR genes profiling data. (b) Multivariate cox regression analysis of the 18 DDR genes expression data. *P* < 0.05 was considered statistically significant in the group.

**Figure 2:** DDR gene signature predicts survival rate of patients with OS patients. (a) Kaplan–Meier survival curves divided OS patients into the high-risk group and low-risk group using the DDR genes signature in the TARGET groups. (b) Area under the curve (AUC) of receiver and the operating characteristic (ROC) curve to assess the sensitivity and specificity of the prognostic model. (c) DDR gene signature was validated in the relapse group. (d) DDR gene signature was validated in the GSE21257 group.

**Figure 3:** The DDR gene signature of independent prognostic factors and developed nomogram. (a) The signature-combined clinical information was used for multivariate cox regression analysis to study the correlation of prognosis of LUSC patients in the training group. (b) Nomogram-combined methylated gene sites signature and clinical‐related variables predict patients' prognosis.

**Figure 4:** Functional analysis of the signature genes. (a) The results of GO analysis. (b) The results of KEGG analysis.

## Data Availability

All the data used to support the findings of this study are included within the article.

## Supplementary Materials

Supplementary Materials Table S1: DDR genes of univariate cox regression analysis in the TARGET group. Table S2: the risk score of DDR gene signature in the TARGET group.
